# Artificial Intelligence System Detection in English Teaching Based on Heuristic Genetic Algorithm

**DOI:** 10.1155/2022/3082779

**Published:** 2022-08-12

**Authors:** Jingwei Tang, Yi Deng

**Affiliations:** ^1^Chongqing Technology and Business University, Chongqing, China; ^2^Assumption University, Bangkok, Thailand; ^3^Chongqing Normal University, Chongqing, China

## Abstract

Using the traditional English teaching mode is difficult to help correct students, and it is difficult to achieve human-computer interaction in oral English communication. In order to improve the effect of English detection and improve teaching efficiency, this article builds an artificial intelligence-assisted teaching system suitable for English teaching based on heuristic genetic algorithms. Furthermore, this article extends the multioffspring genetic algorithm, improves the offspring generation method, and proposes GMOGA, which makes the choice of the number of offspring more flexible. At the same time, it also enables the value of the number of children of the algorithm to be a value that cannot be obtained by the previous algorithm, which further improves the efficiency of the algorithm. In addition, this article combines the actual needs to construct the functional structure of the artificial intelligence system and designs two sets of comparative experiments to verify and analyze the model's performance. The research results show that the model constructed in this article meets the multifunctional requirements of the system and can be applied to practice.

## 1. Introduction

Nowadays, the student evaluation of college English teaching in many universities adopts a combination of formative assessment and summative assessment [1]. Formative assessment includes class attendance, class participation, homework, group learning results , etc. The statistics of the number of participants and each performance are generally recorded with the help of the teacher or learning committee. At the end of the study period, when the total score of the student's test scores is to be counted, teachers find it difficult to calculate the corresponding usual scores for each student fairly. Therefore, they often score based on impressions or take random scores. Obviously, such an evaluation makes it difficult to improve the learning enthusiasm of learning and is not conducive to the development of teacher-classroom interaction [2].

In the discussion of interactive activities in English classroom teaching, some scholars believe that objectively, a good interaction situation can ensure the effectiveness of classroom interaction, and the reason for failure of interaction is mainly reflected in the subjective aspect [3]. For example, students are usually afraid to raise their hands to speak because of their timidity. In the discussion of interactive situations, we also noticed that whether it is students' spontaneous interactive needs or those generated by teachers' guidance, the process invariably reflects the randomness of students' interactive desires. Some scholars also believe that English vocabulary learning plays an important role in English teaching [4]. One of the main reasons for this formulation is that, based on the current general teaching situation in our country, English learners are unlikely to get the same contextual and semantic support as foreign learners in their mother tongue [5].

The English classroom assistant hopes to provide a complete set of solutions to improve the initiative and creativity of learners in traditional English classrooms and help teachers play a leading role in guiding and enlightening [6]. Among them, the blackboard interactive assistant allows learners to interact with the teacher in the classroom “still in place,” thereby helping them overcome the tension of classroom speech. The translation and dictionary modules can provide more timely teaching guidance and ensure the effectiveness of vocabulary learning. In addition, the communication and discussion assistants provide technical guarantee for learner communication, and play an active role in promoting collaboration and jointly accomplishing learning goals [7].

## 2. Related Work

The algorithm proposed in the literature examines all elements in the power set of the conditional attribute set, so it has exponential time complexity [8]. This algorithm has strong theoretical guiding significance, but its calculation speed is slow and it is not easy to be realized by a computer. Therefore, its practical application is very limited. The literature proposed an attribute reduction method of the discernibility matrix, which is an advantageous tool for finding the minimum reduction [9]. It first obtains the core attribute through the discrimination matrix and then finds the minimum disjunctive normal form of the discrimination function according to the core attribute, and finally obtains each disjunctive component of the discrimination function, which corresponds to a reduction. The literature seeks for attribute reduction based on genetic algorithms and through heuristic information such as attribute importance or attribute frequency in a discrimination matrix [10]. Most of the existing literature on attribute reduction is based on two algorithms based on attribute importance and a discrimination matrix. In addition, the algorithm for minimum attribute reduction based on genetic algorithms (referred to as the genetic reduction algorithm) proposed in the reference has also achieved better results [11]. The literature proposed a heuristic genetic algorithm that uses attribute importance as reduction of heuristic information to improve the performance of the algorithm on the basis of optimizing the initial population [12]. The literature proposes a method for generating test sequences based on UML state diagrams using ant colony optimization algorithms [13]. First, the state diagram is converted into a directed graph, and then a group of ants cooperate to explore and generate test sequences on the directed graph. The literature proposed using genetic algorithms to generate test scenarios and optimize them [14]. First, it converts the activity graph to CFG and uses CFG's decision node to randomly generate an initial population. The fitness value of each chromosome is calculated using the basic information flow model and the stack-based weight assignment method. Then, it uses genetic operations to generate test cases and finally selects the test case with the highest fitness value as the test object.

## 3. Algorithm Analysis and Model Building

### 3.1. Basic Genetic Algorithm

The coding method determines the arrangement of genes in the chromosome, which is an important step in the design of genetic algorithms and has an important influence on the performance of genetic algorithms. Binary encoding is an encoding method that maps genes from a search space to binary strings.

(1) $$\begin{array}{c} y=f\left(x\right),x\in \left[a,b\right]. \end{array}$$

Taking the optimal solution of the above formula as an example, the search space is the search interval [*a*, *b*] of *X*. If the encoding length is set to *L*, the encoding problem is transformed into mapping the real number of [*a*, *b*] to an L-bit binary number. Since the genetic algorithm only encodes before initializing the population, the binary encoding does not need to actually convert a certain real value into the corresponding binary value, but determines a coding method and corresponding relationship. In the subsequent algorithm, the population is initialized according to this coding method, and decoding is performed according to the corresponding relationship.

Corresponding to encoding, decoding can map L-bit binary numbers to a real number of [*a*, *b*], which is completed by the following two steps:

(1) The method of converting a binary string *c*_*L*_*c*_*L*−1_ ⋯ *c*_0_ into a corresponding decimal number is as follows:
  (2) $$\begin{array}{c} {\left(c_{L}c_{L-1}\cdots c_{0}\right)}_{2}={\left(\sum {}_{i=0}^{L}c_{i}\times 2^{i}\right)}_{10}=x^{\prime }. \end{array}$$
(2) The real numbers in the interval [*a*, *b*] corresponding to *x*′ are shown in the following formula:
  (3) $$\begin{array}{c} x=a+x^{\prime }\times \frac{b-a}{2^{L}-1}. \end{array}$$

Before calculating the fitness function, we need to sort the individuals in the population. According to the solution requirements, the better solutions are ranked first, and the poorer solutions are ranked last. The fitness function is shown in the following formula:

(4) $$\begin{array}{c} F\left(x_{i}\right)=\frac{N-i+1}{N},i=1,2,\cdots ,N. \end{array}$$

In the above formula, *x*_*i*_ is the sorted individual and *i* is the serial number.

It can be seen from the above formula that the fitness function based on the order satisfies the nonnegative condition and does not rely on any prior knowledge, so it is highly versatile. In addition, the fitness value and the serial number are in a linear relationship, which avoids the phenomenon in some extreme cases, where, because some individuals are particularly good, the probability of other individuals being selected is too low.

The genetic algorithm embodies Darwin's principle of survival of the fittest through selection operations. This article adopts the roulette selection method, sets the population size to *N*, and the operation steps of the roulette method are as follows:

(1) According to the individual fitness value *F*(*x*_*i*_), the algorithm calculates the total fitness *F*_*s*_ of the population. The formula is as follows:
  (5) $$\begin{array}{c} F_{s}=\sum {}_{i=1}^{N}F\left(x_{i}\right). \end{array}$$
(2) The algorithm generates a random number on [0, *F*_*s*_].
(3) The algorithm starts with the first individual and accumulates its fitness until the accumulated fitness exceeds *F*_*s*_. The last individual accumulated is the selected individual.

Gene recombination is an important step in the genetic process of organisms. The crossover operation simulates this genetic operation and is one of the core steps of the genetic algorithm. The crossover methods suitable for binary coding mainly include single-point crossover, two-point crossover, and multipoint crossover.

Single-point crossover, also called simple crossover, is the most basic crossover method. Single-point crossover first randomly generates a crossover point and then exchanges the two parts of the chromosome before and after the crossover point. If the individual code length is *L*, there are *L* − 1 cross points that can be selected. When the given crossover probability *p*_*c*_ is met, it performs a crossover operation to generate two new offspring individuals. The single-point crossover is shown in Figure 1.

The crossover operation can only perform gene recombination between the existing patterns in the population and cannot do anything about the patterns that are not in the population. The mutation operator can perform random search in the neighborhood of the existing pattern of the population, which can effectively expand the search range of the population so that the population can search around the existing pattern and enhance the search ability of the algorithm. In addition, with the increase of the number of iterations, under the action of the selection operator and the crossover operator, the good models are retained, the inferior models are eliminated, and the population diversity decreases. Therefore, mutation operators can effectively enhance population diversity.

Basic bit mutation is to mutate each gene of individual chromosomes with a mutation probability *p*_*m*_, and generate a random number *r*_*i*_ ∈ (0,1), *i*=1,2, ⋯, *L* for each gene. If the random number corresponding to a certain gene is less than the mutation probability, the mutation operation is performed on it; otherwise, the gene value remains unchanged without the mutation operation. Taking binary coding as an example, we set an individual chromosome string as *s*=*a*_1_*a*_2_ ⋯ *a*_*L*_, *a*_*i*_ ∈ (0,1), and the implementation method of mutation operation is as follows:

(1) The probability of mutation *p*_*c*_ is given.
(2) A random number *r*_*i*_ ∈ (0,1), *i*=1,2, ⋯, *L* is generated for each gene.
(3) According to the following formula, a new individual *s*′=*a*_1_'*a*_2_'⋯*a*_*L*_' is generated.
  (6) $$\begin{array}{c} a_{1}^{\prime }=\left\{\begin{array}{cc} 1-a_{i} & r_{i}\leq p_{m}\\ a_{i} & otherwise \end{array}\right\}i\in \left\{0,1,\cdots ,L\right\}. \end{array}$$

Genetic algorithm is an iterative and step-by-step search method. Through multiple iterations of genetic operations, the individuals in the population gradually approach the optimal solution. For complex optimization problems, it takes too long to find the optimal solution, and the algorithm may even converge to a local optimal solution but cannot find the global optimal solution. Therefore, we need to set the stopping conditions for the algorithm, let the algorithm terminate the operation under certain conditions, and output the best individual in the current population as the suboptimal solution. Generally, there are several ways to terminate the iterative process of genetic algorithm:

#### 3.1.1. Operation Time Stop Strategy

This method is to artificially set a maximum algebra in advance. When the population evolves to the maximum algebra or the calculation time reaches the maximum time, the algorithm stops. The disadvantage is that setting selection is difficult, which is not conducive to the generation of optimal solutions, but the evolution can be stopped within a certain period of time.

#### 3.1.2. Solution Accuracy Stop Strategy

This stopping strategy is only suitable for problems with known optimal solutions. When the absolute value of the difference between the optimal individual in the population and the optimal solution of the objective function is less than or equal to a given solution accuracy *ε*, the algorithm terminates. The mathematical expression of the stop strategy is shown in the following formula:

(7) $$\begin{array}{c} \left|f\left(x_{best}^{t}\right)-f^{*}\left(x\right)\right|\leq \varepsilon . \end{array}$$

In the formula, *x*_*best*_^*t*^ is the optimal individual in the *t*-th generation population and *f*^*∗*^(*x*) is the optimal solution to the objective function.

#### 3.1.3. Hybrid Stop Strategy

This method combines two stopping strategies; that is, when the solution accuracy is less than the set value, the algorithm stops; otherwise, the algorithm will continue to run until the number of iterations exceeds the set value.

This article adopts a mixed stop strategy. When the solution accuracy is less than the set value (depending on the function characteristics), the algorithm stops; otherwise, the algorithm will continue to run. When the number of iterations reaches 1000, it stops.

### 3.2. Multichild Genetic Algorithm

One of the branches of mathematical ecology is the study of changes in the size of biological populations over a long period of time. In order to explain the probability that any population can exist for a long time, it is necessary to study its counterproposition, that is, the probability of extinction in a period of time. We assume that there is only one individual. At a later time *t*, the probability of the death of this individual is given by the following formula:

(8) $$\begin{array}{c} p_{0}\left(t|N=1\right)=\frac{\mu e^{\left(\lambda -\mu \right)}-\mu }{\lambda e^{\left(\lambda -\mu \right)t}-\mu }. \end{array}$$

In the above formula, *N* is the population size, *μ* is the mortality rate, and *λ* is the birth rate.

If a population with a population size of *N* is extinct, all *N* individuals in the population will be extinct. The probability of this event is shown in the following equation:

(9) $$\begin{array}{c} p_{0}\left(t\right)={\left[p_{0}\left(t|N=1\right)\right]}^{N}={\left[\frac{\mu e^{\left(\lambda -\mu \right)t}-\mu }{\lambda e^{\left(\lambda -\mu \right)t}-\mu }\right]}^{N}. \end{array}$$

When *t*⟶*∞*, the above formula represents the probability of the final extinction of the population. According to the relationship between *μ* and *λ*, we discuss three situations:

(1) When *λ* < *μ*, the population size grows negatively.
In the above formula, the exponential terms of the numerator and denominator become 0 with *t*⟶*∞*, and the above formula becomes
  (10) $$\begin{array}{c} \underset{t⟶\infty }{\lim}p_{0}\left(t\right)=1\text{.} \end{array}$$
The probability of population extinction is 1, which indicates that the extinction of the population is an inevitable event. Obviously, the population with negative growth in population size will quickly die out.
(2) When *λ* > *μ*, the population size is increasing.
Then, when *t*⟶*∞*, the formula (9) can be transformed into
  (11) $$\begin{array}{c} \underset{t⟶\infty }{\lim}p_{0}\left(t\right)=\underset{t⟶\infty }{\lim}{\left(\frac{\mu e^{\left(\lambda -\mu \right)t}}{\lambda e^{\left(\lambda -\mu \right)t}}\right)}^{N}=\underset{t⟶\infty }{\lim}{\left(\frac{\mu }{\lambda }\right)}^{N}. \end{array}$$
The population has a certain probability of extinction. In this case, the greater the ratio of birth rate to mortality, the larger the population size, the smaller the population extinction probability, and the greater the survival probability.
(3) When *λ*=*μ*, the population size remains unchanged.

The exponent of the exponential term of the numerator and denominator in formula (9) becomes 0 with *t*⟶*∞*, that is, the exponent term becomes 1. At this time, formula (9) becomes

(12) $$\begin{array}{c} \underset{t⟶\infty }{\lim}p_{0}\left(t\right)=1. \end{array}$$

In summary, when *λ*=*μ*, although theoretically the population size will remain unchanged, the population will eventually become extinct. Only when *λ* > *μ*, that is, the population growth rate is positive can the population survive, and the probability of population survival is proportional to the initial population size and the ratio of birth rate to death rate. The research of mathematical ecology has proved the following conclusion: if the initial population size is known, the probability distribution of population size is only related to the product of individual growth rate and time. Therefore, as long as the product of individual growth rate and time is equal, the population will evolve for a shorter time with a high individual growth rate and for a longer time with a low individual growth rate, and the same results will be obtained. Therefore, in order to obtain better individuals in a shorter period of time, it is a better plan to increase the population growth rate.

Algorithm implementation: the single-point crossover multiple generation genetic algorithm (SCMOGA) introduces a new parameter, namely, the number 2*α* of children (*α* is a positive integer greater than 1). We take as an example that every two parent individuals produce 4 offspring (*α*=2). We suppose that the two parent individuals selected to participate in the crossover operation are *P*_1_ and *P*_2_. When *α* crossover points are randomly generated, the chromosomes of *P*_1_ and *P*_2_ are divided into *α*+1 segments, namely, *P*_1_=*A*_1_*B*_1_*C*_1_ and *P*_2_=*A*_2_*B*_2_*C*_2_. The method for generating single-point crossover multiple progenies is as follows: first, it regards the two sides of the first crossover point as two substrings. The first exchange is to exchange the two substrings *B*_1_*C*_1_ and *B*_2_*C*_2_ on the right side of the first intersection to obtain two offspring *O*_1_=*A*_1_*B*_2_*C*_2_ and *O*_2_=*A*_2_*B*_1_*C*_1_. After that, it regards the two sides of the second intersection as two substrings, respectively. The second exchange is to exchange the two substrings *C*_1_ and *C*_2_ on the right side of the second intersection to obtain two offspring *O*_3_=*A*_1_*B*_1_*C*_2_ and *O*_4_=*A*_2_*B*_2_*C*_1_. The individual generation method of SCMOGA progeny can be shown in Figure 2.

It can be seen that the number of new offspring individuals generated by SCMOGA will greatly increase, which can increase the possibility of producing better individuals and can greatly improve the performance of the single-point crossover genetic algorithm. The larger the value of *α*, the greater the number of offspring produced in each iteration, the faster the population evolution speed, and the fewer the iterations required for convergence. At the same time, as the value of *α* increases, the more calculations per iteration, the more time each iteration consumes. Therefore, finding a compromise *α* value that minimizes the total solution time has a great impact on the performance of the algorithm. At present, there is no relevant research to guide the selection of *α* value.

## 4. Intraspecific Competition Operation

If the number of offspring obtained by SCMOGA through the crossover operation is *αN* (crossover probability *P*_*c*_ is 1), then the total number of offspring individuals at this time is *N*_1_=*αN*. When *N*_1_ offspring are added to *E* elite individuals retained by the parent, the number of individuals in the temporary population is *N*_1_=*αN*+*E* and *N*_1_ > *N*. Therefore, the number of offspring individuals produced by SCMOGA far exceeds the initial population size. Therefore, to keep the population size constant during each iteration, it is necessary to retain *N* outstanding individuals among *N*_1_ individuals to form a progeny population, which ensures the stability of the population size. We call this operation an intraspecies competition.

SCMOGA produces more offspring individuals per crossover than the traditional single-point crossover genetic algorithm. In addition to competition between individuals and the environment, it introduces intraspecific competition operations to force individuals within the population compete with each other. In this fierce competition, the individuals who can survive are excellent individuals, and some poor individuals are eliminated because they cannot adapt to this fierce competition, so that the population develops in a better direction.

The basic VRP can be described as follows: it first plans an evolutionary route based on a given series of information, and then the particles start from the center point, visit each node for English detection, and finally return to the center point. In this process, the requirements can not only meet the requirements of English testing and other constraints but also minimize testing costs. A schematic diagram of the particle path problem is shown in Figure 3. The box in the center of the graph represents the origin of the delivery tool, the small circle represents the English detection node to be visited, and the line segment between the nodes represents the delivery path. In order to describe VRP with mathematical symbols, the symbols are now defined as follows:

*M*: number of particles used.
*d*_*i*_: demand for English test point *i*.
*C*_*ij*_: distribution cost incurred by particles visiting arc (*i*, *j*).
*N*: number of nodes.
*C*: maximum load of particles.
*C*_*v*_: maximum number of particles available.
*U*_*i*_: the particle is the minimum detection amount required to serve node *i* and the nodes before it.
  (13) $$\begin{array}{c} x_{ij}=\left\{\begin{array}{cc} 1 & There\;is\;vehicle\;access\;arc\left(i,j\right),\\ 0 & otherwise. \end{array}\right. \end{array}$$

The hierarchical objective function of the VRP mathematical model is constructed. We take the least amount of particles used as the first-level goal and the lowest particle delivery cost as the second-level goal, and define its objective function as the formula:

(14) $$\begin{array}{c} \min F=p_{1}M+p_{2}\sum {}_{i=0}^{N}\sum {}_{j=0}^{N}C_{ij}x_{ij}. \end{array}$$

In the formula, *F* represents the objective function, *p*_1_, *p*_2_ is an integer, and *p*_1_ ≥ *p*_2_. The purpose of introducing the parameter *p*_1_, *p*_2_ in the objective function is to ensure that in the process of solving, the least amount of particles is used as the first optimization goal and the lowest particle delivery cost is used as the secondary optimization goal.

(15) $$\begin{array}{c} x_{ii}=0,i=1,2,\cdots ,N, \end{array}$$

(16) $$\begin{array}{c} \sum_{i=1}^{N}x_{ij}=1,i=2,3,\cdots ,N, \end{array}$$

(17) $$\begin{array}{c} \sum_{j=1}^{N}x_{ij}=1,i=2,3,\cdots ,N, \end{array}$$

(18) $$\begin{array}{c} U_{i}\leq C,i=2,3,\cdots ,N, \end{array}$$

(19) $$\begin{array}{c} U_{i}\geq U_{j}+d_{i}+C\left(x_{ij}+x_{ji}-1\right)-x_{ij}\left(d_{i}+d_{j}\right) \end{array}$$

(20) $$\begin{array}{c} U_{i}\leq C-\left(C-d_{i}\right)x_{1i},i=2,3,\cdots ,N, \end{array}$$

(21) $$\begin{array}{c} U_{j}\geq d_{j}+\sum_{i=1}^{N}d_{i}x_{ij},j=2,3,\cdots ,N, \end{array}$$

(22) $$\begin{array}{c} M\geq \frac{1}{C}\sum_{i=1}^{N}d_{i}, \end{array}$$

(23) $$\begin{array}{c} \sum {}_{j=1}^{N}x_{1j}=M, \end{array}$$

(24) $$\begin{array}{c} M\leq C_{v}, \end{array}$$

(25) $$\begin{array}{c} x_{ij}=0or1, \end{array}$$

(26) $$\begin{array}{c} M\;is\;an\;integer. \end{array}$$

Equation (15) ensures that particles will not travel from a city to itself; equation (16) ensures that each English test is only served once; constrained (17) ensures that particles only leave each English test once. (18) is the particle load constraint, the loading capacity of all cars does not exceed the particle load *C*; (19) is the detection volume constraint between the front and rear nodes; (20) is the detection volume constraint for the first node; (21) is the detection volume constraint except for the first node; (22) is the minimum required particle number limit; (23) is the minimum dispatched particle number limit; (24) is the maximum particle number limit; (25) is the 0-1 constraint of *x*; (26) indicates that the required number of particles *M* is an integer.

## 5. Simulation Results

### 5.1. Model Building

As shown in Figure 4, the free dialogue in the human-computer interaction system based on English teaching mainly includes speech recognition, language understanding, and dialogue management. Among them, dialogue management refers to integrating the context and historical dialogue content into the dialogue and organizing reasonable response sentences. In most cases, the boundaries between speech understanding and dialogue management are blurred, and they are often studied as a unified whole. The main work of the free dialogue function in this article is the part where the program gives a response after the speech recognition process is executed, which is collectively referred to as dialogue management in the following.

The emotional interaction between artificial intelligence systems and users can be roughly divided into three levels: form, content, and behavior. The emotional interaction of behavior is the core of the design, which runs through the entire interaction design process. Open arm posture, head movement, and gaze following can effectively promote the expression of NAO, which makes users more willing to interact with it. As shown in Figure 5, the interactive behaviors in the emotional interaction of the artificial intelligence system include external actions, facial expressions, and voice emotions. Among them, the emotions of the external actions of the artificial intelligence system can be mainly reflected by body movements and gestures, the facial expressions of the artificial intelligence system can mainly be realized by the brightness changes of the artificial intelligence system's facial LEDs and the head rotation, and the voice emotion of the artificial intelligence system is mainly reflected by the pause of the sentence, the speed, and pitch of the voice In the dialogue process of the artificial intelligence system, external actions, facial expressions, voice emotions, and other parts will cooperate with each other.

In this article, when the learner and the artificial intelligence system have a normal conversation, the environment is stable, and the conversation content involved is limited. In addition, the time required for the artificial intelligence system to be reflected in real-time communication is relatively high. Therefore, in this article, in the speech synthesis process of the artificial intelligence system, keywords representing emotions should be extracted and marked. When the synthetic content corresponding to the keyword is triggered, the action representing the emotion is called to cooperate with it, and the process is shown in Figure 6. The artificial intelligence system receives the user's voice input, calls the voice recognition module, and determines the next voice output content according to the recognition content. If there are keywords representing emotions in the output, the corresponding action in the action library is called and the voice content is output.

### 5.2. System Test

The system constructed in this article can realize intelligent recognition and sentiment analysis of English dialogue. Therefore, in the system test, the voice and emotion are mainly tested, and two sets of experiments are set up for analysis. First of all, this article conducts voice signal detection and sets 96 groups of dialogues for detection. The results are shown in Figure 7.

It can be seen from Figure 7 that the model constructed in this article performs well in voice signal monitoring. Next, this article uses 96 groups of dialogues to perform emotion detection, and the results are shown in Figure 8.

From the above detection results, it can be seen that the model constructed in this article performs very well in emotion and speech detection, so the model constructed in this article meets actual needs.

## 6. Conclusion

The English classroom assistant hopes to provide a comprehensive set of solutions to improve the initiative and creativity of learners in traditional English classrooms and help teachers play a leading role in guiding and enlightening. This article proposes a solution for English classroom assistants based on smart detection. Using the English classroom as an example, this article analyzes, designs, and implements such a set of intelligent English teaching assistants based on the unsatisfied demands of learners in the classroom. In this article, the multioffspring genetic algorithm is extended, the offspring generation method is improved, and GMOGA is proposed, which makes the choice of the number of offspring more flexible. At the same time, it allows the algorithm's number of children to be a value that cannot be obtained by the previous algorithm, which further improves the efficiency of the algorithm. After a long time, this article proposes a VRP model that uses MOGA for solutions, and tests it on a test data set. The test results validate the effectiveness of the VRP model and MOGA. Finally, this article designs a control experiment to verify and analyze the performance of the model. According to the research findings, the model constructed in this article performs very well in emotion and speech detection, so the model constructed in this article meets actual needs.

## Figures and Tables

**Figure 1:** Point cross.

**Figure 2:** Single-point crossover multiple progeny genetic algorithm (*α*=2).

**Figure 3:** Schematic diagram of particle path problem.

**Figure 4:** Free dialogue function group.

**Figure 5:** Emotional interaction behavior of artificial intelligence system.

**Figure 6:** Flow chart of emotional assistance dialogue.

**Figure 7:** Statistical diagram of speech signal detection results.

**Figure 8:** Statistical diagram of speech emotion detection results.

## Data Availability

The data used to support the findings of this study are available from the corresponding author upon request.
